The article "Improved Feature Pyramid Convolutional Neural Network for Effective Recognition of Music Scores" was published in 2022. Journal: Comput Intell Neurosci.

# Improved Feature Pyramid Convolutional Neural Network for Effective Recognition of Music Scores

**DOI:** 10.1155/2022/6071114

**Published:** 2022-05-09

**Authors:** Lei Li

**Affiliations:** College of Music, Handan University, Handan 056005, Hebei Province, China

## Abstract

Music written by composers and performed by multidimensional instruments is an art form that reflects real-life emotions. Historically, people disseminated music primarily through sheet music recording and oral transmission. Among them, recording music in sheet music form was a great musical invention. It became the carrier of music communication and inheritance, as well as a record of humanity's magnificent music culture. The advent of digital technology solves the problem of difficult musical score storage and distribution. However, there are many drawbacks to using data in image format, and extracting music score information in editable form from image data is currently a challenge. An improved convolutional neural network for musical score recognition is proposed in this paper. Because the traditional convolutional neural network SEGNET misclassifies some pixels, this paper employs the feature pyramid structure. Use additional branch paths to fuse shallow image details, shallow texture features that are beneficial to small objects, and high-level features of global information, enrich the multi-scale semantic information of the model, and alleviate the problem of the lack of multiscale semantic information in the model. Poor recognition performance is caused by semantic information. By comparing the recognition effects of other models, the experimental results show that the proposed musical score recognition model has a higher recognition accuracy and a stronger generalization performance. The improved generalization performance allows the musical score recognition method to be applied to more types of musical score recognition scenarios, and such a recognition model has more practical value.

## 1. Introduction

Music is a vital means of cultural dissemination and communication, and as one of its carriers, musical notation is the most direct method of learning, sharing, and disseminating music through the detailed recording of notes and other related information. Many musical scores, on the other hand, have not been published or are only available in paper format. They are easily damaged or even lost as the environment and times change. As a result, the total preservation of paper scores is critical. Scanning or photographing paper scores is generally a preferable way to preserve them, it is easily constrained by factors such as scanning quality and storage capacity. Fast advancements in hardware performance, such as scanners and memory, enable people to retain more and better musical scores, while computers are unable to directly exploit this digitized musical score. Only by extracting the symbolic content from the score image can users make more flexible and convenient use of the score to perform music arrangement, synthesis, and other operations. The advancement of theory and technology in the fields of computer and image processing enables the creation of novel techniques for extracting symbols from musical scores. The resulting Optical Score Recognition (OMR) technology converts printed scores to symbolic scores, such as MIDI files, transforming the optical score image into not just a digital image but also a computer-readable file. This has a substantial and far-reaching effect on the domains of music information retrieval and music-assisted instruction. While commercial recognition software is available, recognition methods continue to suffer from issues such as poor antinoise performance and low recognition accuracy. As a result, it is critical to continue researching OMR algorithms with increased resilience and accuracy.

The article "Improved Feature Pyramid Convolutional Neural Network for Effective Recognition of Music Scores" was published in 2022. Journal: Comput Intell Neurosci.

As can be seen, note recognition is the focal point of musical score recognition, with note recognition emphasizing the characteristic information carried by the correlation between notes. As a result, the identification of musical notes has significant research value as a type of special symbol. Homenda [1] and Rebelo et al. [2] proposed a pattern recognition method for musical notation. Due to deep learning's superior performance in image processing, researchers began to use the neural network models for musical score recognition. Calvo-Zaragoza et al. [3] treated stave detection as a classification task, used CNN to detect staves, labeled each pixel as staves or notes, and trained in pairs using data with and without staves. The experimental results show that the effect is superior to most traditional methods, even when no postprocessing is used. Pinheiro et al. [4] compared CNNs to the classical deep learning networks for note recognition tasks. Rebelo et al. [2] used neural networks for the first time in the note classification stage, comparing them to SVM and other models; while the results were not favorable, they laid the groundwork for future research. Following that, Wen et al. [5] used multilayer perceptron to build the models with different parameters for the two types of notes in order to achieve classification, and the classification effect was enhanced. The CNN model is used in reference [6] for staff deletion and note classification, but the classification effect is unstable. Choi et al. [7] achieved a 99.2 percent accuracy in detecting sharps, flats, and reductions in diacritics using a combination of CNN and Spatial Transformer Networks (STN). The two methods described above are only useful for identifying a specific symbol; their application scope is limited, and their expansion is limited. Reference [8] suggests the use of electronic pen technology and implements the CNN model [9] to convert handwritten musical scores to electronic musical scores. The study's accuracy was insufficient to identify longer and more challenging notes. Tuggener et al. [10] considered the R–CNN for optical score recognition because of its remarkable performance in object detection. To recognize the score image, the ResNet-101 is coupled to the RefineNet upsampling network and integrated with the bounding box detection algorithm. This approach is effective at recognizing entire rests, but it is less than 50% accurate at recognizing other notes, particularly diacritics and time signatures.

The article "Improved Feature Pyramid Convolutional Neural Network for Effective Recognition of Music Scores" was published in 2022. Journal: Comput Intell Neurosci.

The study mentioned above have achieved some progress in their disciplines, but there are still certain issues, as listed below. For example, in a machine-learning-based recognition process, different features must be selected, and there is currently no standard feature extraction approach. Furthermore, the note sequence in the dataset is merely a collection of simple notes with insufficient richness and diversity, making the model's generalization ability low and prone to overfitting. Furthermore, because the data set is relatively clean, the algorithm will be less robust, and the recognition accuracy of noisy and distorted sheet music images will be much lower. This study uses a deep learning model to solve the problem of feature selection, avoiding the need to select feature selection strategies. This research provides an updated SEGNET model for music score recognition with the goal of improving generalization. The revised SEGNET model's main idea is to take the feature pyramid structure from SEGNET [11, 12]. Use additional branch paths to fuse image details from shallow layers, shallow texture features that are beneficial to small objects, and high layer features that fully describe the global information, enriching the model's multiscale semantic information and alleviating the lack of multiscale semantic information. Poor image segmentation is a result of semantic information.

## 2. Knowledge of Music Score Recognition

### 2.1. Score Notation

The origin of the stave symbolizes musicians' unwavering efforts to express their inner musical inspiration through written figures [13]. Musical symbols, like letters in the alphabet, are assigned a distinct musical meaning that intuitively explains the connected properties among various sounds, such as pitch, beat, time duration [14].  Figure 1 shows a selection of scanned musical score images. The staves are the most important part of the musical score in the illustration, and other musical symbols are evenly arranged on five parallel lines. The following are some of the musical symbols utilized in this work. The staff is made up of five lines that are parallel to each other and four spaces among them. As seen in Figure 1, lower and upper lines are occasionally used as needed. As seen in Figure 2, musical symbols are placed on a line or in an interval to indicate different pitches.

The article "Improved Feature Pyramid Convolutional Neural Network for Effective Recognition of Music Scores" was published in 2022. Journal: Comput Intell Neurosci.

The clef, which is usually found at the far left of the staff line, is used to determine the pitch of the staff. The treble clef, bass clef, and tenor clef are the most used clefs [15]. A note is a symbol that indicates how far a note has progressed. A note is made up of three parts: a note head, a note stem, and a note tail. Different notes represent different lengths of time.  Table 1 shows the different types of notes.

### 2.2. Music Score Image Features

Due to the wide variety of musical notation, this presents a challenge for score recognition. Note objects vary in size and shape, especially in handwritten scores and making music extraction more complicated and difficult. Different authors write the same flat, treble clef, and eighth note, but their symbols are quite different and making identification difficult. The following characteristics of sheet music images are summarized in this paper:

1. Considering the score image's binary nature: Because most images of musical scores are black and white, researchers can simplify the image information through binarization, which is convenient for subsequent identification. However, selecting the binarization threshold incorrectly will result in the loss of useful information.
2. Musical notation takes many forms, and each note has a rich meaning: The same note has a different sound value when played in different positions. Occasionally, different notes can express the same sound. This wide range of musical notation meaning necessitates a certain musical foundation to be comprehend.
3. The images on sheet music are associative: Superimposed spectral lines and symbols are interleaved and glued together. Keeping the staff line is not conducive to extracting the note object, and deleting the staff line is very likely to result in the deletion phenomenon, which makes the note image incomplete. Not only are notes related to staves, but they are also related to one another.
4. Musical notation binding: The score image contains some implicit constraint information, for example, if the clef is a treble staff, the musical meanings of notes at different positions should be read in accordance with the treble staff's corresponding pitch values. Another example is that the score's time signature should be equal to the number in the bar. Sheet music images contain a wealth of musical background knowledge. This necessitates users establishing the overall relationship from a macro perspective as well as understanding the meaning of each note from a microperspective. Only in this manner it is possible to reconstruct musical semantics. However, the interdisciplinary span is broad, which has made identifying musical scores difficult.

The article "Improved Feature Pyramid Convolutional Neural Network for Effective Recognition of Music Scores" was published in 2022. Journal: Comput Intell Neurosci.

## 3. Improved Convolutional Neural Network for Music Score Recognition

### 3.1. The Music Score Recognition Process Based on Neural Network

Figure 3 depicts the neural network-based music score recognition process. The entire score recognition process is divided into seven stages: acquiring data, creating a data set, preprocessing data, designing a network, training the network, evaluating the network, and determining the recognition result. Because the goal of this study is to train a deep learning network for score recognition, the corresponding score image data must be first obtained. Following the acquisition of music data, a music data set is created in accordance with the standard. Perform some preprocessing operations on the data input into the network after creating the dataset, such as data augmentation. When the data are ready, the score recognition network is designed using the various neural network layers. Following the construction of the corresponding music score recognition network, the corresponding deep learning framework must be used to train the network. The loop operation is used in the specific training scheme to continuously perform iterative tuning until a satisfactory result is obtained or the set number of iterations is reached. The training result will eventually be saved as a model file after network training. The corresponding metrics can be used to evaluate the performance of the network in order to verify its performance, and the final model can be used for musical score recognition.

### 3.2. SEGNET Model

SEGNET is a classic deep learning segmentation network, which is a fully convolutional neural network. Its network structure is shown in Figure 4.

This is an encoder-decoder model, and the SEGNET model has no exception. Convolution, BN, RELU activation, and pooling operations are continuously superimposed in the encoder stage. Using a continual superposition of convolution operations, the encoder's receptive field expands to automatically identify valuable characteristics in the input image. Upsampling, convolution, BN, and RELU activation functions are all layered on top of each other in the decoder stage. After boosting the feature map's size with an upsampling operation, the convolution operation is used to remove any noise that may have been introduced by the upsampling.

The article "Improved Feature Pyramid Convolutional Neural Network for Effective Recognition of Music Scores" was published in 2022. Journal: Comput Intell Neurosci.

SEGNET's upsampling process is distinct from those of the FCN [16] and UNET [17]. As a result of this, SEGNET keeps residual information from the previous pooling layer in order to maintain the original location of the target edge in the image throughout the encoder stage. This information is utilized as a supplement in the decoder step. Upsample the feature map in accordance with the given index information, then restore it to its original size by assigning the feature map value to its original place and assigning 0 to all other positions. In the convolution operation, the upsampled feature map is manipulated to decrease the noise caused by the upsampling procedure. Upsampling results are smoothed and denoised using convolution kernel parameters that are constantly updated in response to the gradient in the data set. The model returns predictions of the same size as the original input in the final convolutional phase of the model. Additional channels equal to the number of categories are included in the prediction result. Using the softmax function, it is possible to forecast the category of each pixel. Loss functions for training models are based on cross-entropy, and the model parameters are adjusted by the backpropagation in order to minimize this loss in the training phase. As a result, the SEGNET model is not optimal for image segmentation during testing, despite its great improvement over FCN. Smaller objects are overlooked during segmentation in the SEGNET model because of the behavior described above. For the most part, this is because the SEGNET model makes use of only a small subset of available multiscale semantic data. Each decoder just makes use of the pooling index that has been supplied to it. Pixel classification is not possible with this model because it does not consider the pixel as a whole. Each pixel's semantic and texture information limits the categorization accuracy of that pixel.

### 3.3. Improved SEGNET Network

By performing convolution and pooling operations on the features output from the high-level, the feature maps obtained by successive stacking have greater fusion in the multilayer neural network model. This part of the features is more inclined to describe the global context information. Because the convolution and pooling operations are stacked less in the lower layers of the network model, the detailed texture information is lost less, and most of the original image details, including the image's edges and textures, are retained in this part of the features.

The article "Improved Feature Pyramid Convolutional Neural Network for Effective Recognition of Music Scores" was published in 2022. Journal: Comput Intell Neurosci.

This paper applies the concept of feature pyramid structure to the problem of misclassification of some pixels in SEGNET and uses additional branch paths to describe image details from its shallow layers, as well as shallow texture features that are beneficial to small targets compared to those from high layers. The features that have sufficient global information descriptions are fused to enrich the model's multiscale semantic information and alleviate the problem of poor segmentation caused by a lack of multiscale semantic information. We have specifically improved the SEGNET model structure as follows: First, the features of each encoder layer are fused using bottom-up pathways and horizontal connections to produce features with multiscale semantic information. The feature is then sent to the decoder for the subsequent convolution operation. Given that the operation of upsampling the feature map will inevitably introduce noise, we keep a portion of the SEGNET decoder's original structure. A convolution operation is added after each upsampling operation to filter the features and reduce the noise effect caused by the upsampling. Furthermore, due to fewer convolution operations, there is still a lot of redundant information in the features of SEGNET's first layer. When the features are integrated, the features of the first layer are not included to avoid introducing additional parameters and to ensure the inference time.

Second, we do not use the common concatenate operation in feature fusion. The reason for this is that the concatenate operation increases the number of channels in the convolutional layer input. A large increase in the number of channels in the case of the same size convolution kernel will result in additional computational burden. This influences the model's actual inference speed. The integration method used in the Feature Pyramid Network is chosen in this paper. The first step for the two feature maps that must be integrated uses an upsampling operation to adjust the smaller size feature map to ensure that it is the same size as the larger feature map. The second step uses 1 × 1 convolutions to align the channel numbers of the two feature maps. Finally, the integration is completed by incorporating the corresponding position elements onto the feature map. In comparison to the concatenate operation, the corresponding element completes the function of multiscale semantic information integration while increasing the number of parameters to a minimum.

The article "Improved Feature Pyramid Convolutional Neural Network for Effective Recognition of Music Scores" was published in 2022. Journal: Comput Intell Neurosci.

As shown in Figure 5, the improved SEGNET network's input source in the decoder part is divided into two parts: the features of the previous layer and the features after integrating multiscale semantic information passed through lateral connections. The type and quantity of information contained in the encoder part has improved when compared to only using the pooling index and the previous layer features. Because the shallowest layer's features are too close to the input and there are fewer convolution kernels here, there is still more noise in the features, so this part of the features is not used for the final prediction.

### 3.4. The Optimization Goal of Improving the Network

In this research, the multiclass cross-entropy is used as the model's optimization goal in the training phase for a single batch:

(1) $$\begin{array}{c} L_{ce}=-\frac{1}{N}\sum_{i=1}^{N}\sum_{j}^{M}y_{j}\log\left(p_{j}\right), \end{array}$$

where *y*_*j*_ is the category label associated with the pixel, *p*_*j*_ is the predicted probability output by the deep learning model, and *M* is the number of pixels in each image. During the actual training process, images of varying sizes will be unified by upsampling or downsampling operations to unify the image input size, where *N* represents the number of samples included in the batch, and each sample in each batch contributes the same amount to the loss.

Batch normalization and L2 regularization are used during the model construction process to prevent overfitting. Batch normalization is placed in the model after a convolutional layer and before the activation layer. Batch normalization increases the model's convergence speed, ensures the stability of the model training process, and eliminates jitter and oscillation of the loss curve. Furthermore, the additional L2 regularization term on the loss function term avoids the numerical issues that arise during the model parameter updating process. The loss function of the final model is

(2) $$\begin{array}{c} L=L_{ce}+\alpha L_{\text{regular}}, \end{array}$$

where *α* is a parameter used to adjust the effect of L2 regularization on the loss function, and *L*_*regular*_ is

(3) $$\begin{array}{c} L_{\text{regular}}=\sum w_{i}^{2}, \end{array}$$

where *w*_*i*_^2^ is the parameter's second-order norm when the parameter is set too high, it has an effect on the loss function's value. Because the model's goal is to minimize (3), the parameter floating range will be limited to ensure that it is not too large, reducing the risk of model overfitting.

### 3.5. Model Training

In the training phase of the model, exponential sliding decay is used as follows:

(4) $$\begin{array}{c} LR=LR_{\text{current}}*LR\_{\text{decay}}^{t_{\text{global}}/s_{\text{decay}}}, \end{array}$$

where *LR*_current_ denotes the current learning rate, *t*_global_ denotes the number of global iterations, and *s*_decay_ denotes the decay step size on the training set, each batch of 5 images is fully iterated 10 times, the learning rate is set to 0.01, the decay index is set to 0.95, and the decay step size is set to 100. This paper compared three optimizers during the model training process: mini-Batch SGD, Mini-Batch Momentum SGD, and Adam, an adaptive optimization algorithm. The experimental results show that when the momentum coefficient is set to 0.92, the performance of the Mini-Batch Momentum SGD is optimal.

The article "Improved Feature Pyramid Convolutional Neural Network for Effective Recognition of Music Scores" was published in 2022. Journal: Comput Intell Neurosci.

## 4. Experimental Verification and Analysis

### 4.1. Experimental Basic Settings

The Universal Music Symbol Collection dataset is used in this paper, which combines 7 datasets into a large dataset of 90,000 tiny music symbol images from 79 categories that can be used to train a universal music symbol classifier. 74,000 symbols are handwritten, while 16,000 are printed. Most of the notation examples include not only the arrangement and combination of simple note sequences but also a broader range of notes such as clefs, time signatures, sharps and falls, rests, and difficult notes to recognize such as arpeggione and dotted notes. During the experiment, the data set was divided into training and test sets in an 8 : 2 ratio.

This paper's experimental environment includes the Ubuntu15.10 operating system, an Intel Core i7-6700 CPU, 12 GB of running memory, an Nvidia GTX1080Ti GPU, and the TensorFlow deep learning framework. Accuracy, precision, recall, specificity, and G-mean are the evaluation indicators used in this paper.

(5) $$\begin{array}{c} \text{Accuracy}=\frac{a+b}{a+c+d+b},\\ \text{Precision}=\frac{a}{a+c},\\ \text{Recall}=\frac{a}{a+d},\\ \text{Specificity}=\frac{b}{b+c},\\ G-\text{mean}=\sqrt{\text{Recall}*\text{Specificity}}, \end{array}$$

*a* denotes the number of symbols correctly detected as belonging to a positive class, implying that it is both positive and the classification result is also positive. *c* is the symbol for the false positive class, which means that it was initially negative but now has a positive classification result. *d* is the number of falsely negative signs; that is, otherwise positive signs that are mistakenly interpreted as negative. *b* is the number of negative samples that were correctly excluded.

### 4.2. Experimental Results and Analysis

Reference [18], Reference [19], Reference [20], SEGNET [21], and improved SEGNET were utilized as comparison algorithms.  Table 2 shows the experimental results.  Figure 6 shows the comparison of each indicator under different methods.

The article "Improved Feature Pyramid Convolutional Neural Network for Effective Recognition of Music Scores" was published in 2022. Journal: Comput Intell Neurosci.

Because the algorithm model utilized in this study is susceptible to noise and has weak anti-interference, the accuracy rate and other index values reported in reference [18] are all low in Table 2, resulting in extremely low recognition accuracy for multivoice musical notes. Reference [19] employs a deep watershed detector for music score recognition, and the results are better than reference [18]. Furthermore, reference [18] requires cutting the music score image into a single staff image for input, which significantly increases system runtime. Reference [20] uses region-based convolutional neural networks to recognize musical scores, and the addition of deep learning models dramatically increases musical score identification performance. In terms of accuracy, precision, recall, specificity, and G-mean, reference [20] has improved by 10.79 percent, 10.61 percent, 12.31 percent, 10.65 percent, and 11.49 percent, respectively, over reference [18]. However, this study's model can only learn local information, which has an impact on the overall recognition effect, the SEGNET model's experimental effect is similar to that of the reference [20], and the recognition rate advantage is not noticeable. The upgraded SEGNET employed in this work has greatly enhanced score recognition performance. In terms of accuracy, precision, recall, specificity, and G-mean, it has improved by 2.59 percent, 1.04 percent, 2.93 percent, 1.7 percent, and 2.33 percent, respectively, as compared to reference [20] with the best effect in the comparison experiment.

The comparative models used traditional convolutional neural network (CNN) [22], recurrent neural network (RNN) [23], fully convolutional network (FCN) [24], and SEGNET to validate this study's outstanding performance in terms of model training speed.  Table 3 shows the obtained recognition results, and Table 4 shows the training time for each model.

It can be seen from the experimental data presented in Table 3 and Figure 7 that the performance of the deep learning model in recognizing musical scores is good. CNN surpasses RNN in terms of performance when comparing different deep learning models. The FCN model exhibits a strong recognition effect when compared to the convolutional neural network model. Overall, the performance of this model in terms of score recognition is marginally worse than that of the modified SEGNET model provided in this study. However, the disparity between the two models is not significant. To summarize, among the numerous deep learning models available, the performance increase of the model suggested in this research is not immediately apparent, as evidenced by the recognition accuracy rate obtained using the model.

The article "Improved Feature Pyramid Convolutional Neural Network for Effective Recognition of Music Scores" was published in 2022. Journal: Comput Intell Neurosci.

Model training times for CNN, RNN, and FCN all surpass 1000 ms, and only SEGNET and the model employed in this paper are within 1000 ms, according to the data in Table 4 and Figure 8. The SEGNET model eliminates the full connection layer in order to improve speed, adds batch normalization in order to speed up convergence and suppress overfitting, adds Bayesian in order to output the uncertainty segmentation value of the image, adds test batch dropout in order to improve performance during testing, and adds batch normalization in order to speed up convergence and suppress overfitting. It is necessary to deal with the unbalanced phenomenon of segmentation samples by employing a weighted softmax algorithm. As a result, the SEGNET model is being used for score recognition in this research, which is one of the justifications for this choice. It can be seen from the experimental data that the improved SEGNET algorithm proposed in this paper basically achieves the expected goal in terms of retaining the advantage of the SEGNET model in training time while also improving the recognition performance of the model, as can be seen from the experimental data.

## 5. Conclusion

Recognizing music scores is a proposal. Technology is at the heart of both the preservation of music data and the creation of contemporary music. The systematic study of musical score recognition has the potential to promote the coordinated development of interdisciplinary subjects such as music, computer science, and artificial intelligence. Combining scientific research with art, on the one hand, contributes to the expansion of the natural sciences' research scope. Technology, on the other hand, is an important factor in promoting the development of art. In the new era, technology has accelerated the development of smart music while also enhancing the brilliance of art. To improve the accuracy, generalization, and stability of musical score recognition while shortening model training time, this paper builds on the idea of SEGNET's feature pyramid structure and uses additional branch paths to describe image details from its shallow layers. The shallow texture features that are beneficial to the target are combined with higher layer features that accurately describe the global information. This can improve the model's multiscale semantic information, thereby resolving the issue of poor image segmentation due to a lack of multiscale information. This paper both theoretically and experimentally validates the superiority and practical utility of the proposed model. However, when confronted with unbalanced data, our model has some limitations. Imbalanced data will significantly reduce the proposed model's recognition performance. When confronted with an imbalanced data recognition scene, how to maintain the excellent recognition performance of the residence model is a direction that this paper should continue to investigate in the future.

The article "Improved Feature Pyramid Convolutional Neural Network for Effective Recognition of Music Scores" was published in 2022. Journal: Comput Intell Neurosci.

## Figures and Tables

**Figure 1:** Staff table.

**Figure 2:** Treble staff pitch.

**Figure 3:** Music score recognition process.

**Figure 4:** SEGNET network structure.

**Figure 5:** Improved SEGNET network structure.

**Figure 6:** Comparison of music score recognition results across studies.

**Figure 7:** score recognition results for each deep learning model.

**Figure 8:** Training time comparison.

**Table 1:** Types of notes.

Note	Details
Whole note	The hollow white note is the whole note, which is the longest of all notes, and all other notes are based on it.
2nd note	Consisting of a hollow head and stem, it is only half the length of a whole note.
Quarter note	Consisting of a hollow head and stem, it is only half the length of a half note.
8th note	Consisting of a hollow head and stem, it is only half the length of a quarter note.
16th note	Consisting of a hollow head and stem, it is only half the length of an eighth note.

**Table 2:** Identification results of different methods.

Index\Model	Ref. [18]	Ref. [19]	Ref. [20]	SEGNET	Proposed
Accuracy	0.8316	0.8875	0.9214	0.9115	0.9453
Precision	0.8542	0.9088	0.9449	0.9424	0.9547
Recall	0.8074	0.8550	0.9068	0.9102	0.9334
Specificity	0.8523	0.9122	0.9431	0.9455	0.9591
G-mean	0.8294	0.8831	0.9247	0.9277	0.9462

**Table 3:** Music score recognition results of each model.

Index\Model	CNN	RNN	FCN	SEGNET	Proposed
Accuracy	0.9291	0.9054	0.9413	0.9115	0.9453
Precision	0.9332	0.9273	0.9515	0.9424	0.9547
Recall	0.8968	0.8948	0.9317	0.9102	0.9334
Specificity	0.9305	0.9210	0.9598	0.9455	0.9591
G-mean	0.9148	0.9109	0.9415	0.9277	0.9462

**Table 4:** Training time of each model.

Model	CNN	RNN	FCN	SEGNET	Proposed
Time(ms)	1288	1435	1203	532	689

## Data Availability

The labeled dataset used to support the findings of this study are available from the corresponding authors upon request.
